# Source Localization of EEG Brainwaves Activities via Mother Wavelets Families for SWT Decomposition

**DOI:** 10.1155/2021/9938646

**Published:** 2021-04-28

**Authors:** Tarek Frikha, Najmeddine Abdennour, Faten Chaabane, Oussama Ghorbel, Rami Ayedi, Osama R. Shahin, Omar Cheikhrouhou

**Affiliations:** ^1^CES Lab, Université de Sfax, Sfax, Tunisia; ^2^Regim-Lab, Université de Sfax, Sfax 3038, Tunisia; ^3^Jouf University, Sakakah, Saudi Arabia; ^4^College of CIT, Taif University, P.O. Box 11099, Taif 21944, Saudi Arabia

## Abstract

A Brain-Computer Interface (BCI) is a system used to communicate with an external world through the brain activity. The brain activity is measured by electroencephalography (EEG) signal and then processed by a BCI system. EEG source reconstruction could be a way to improve the accuracy of EEG classification in EEG based brain-computer interface (BCI). The source localization of the human brain activities can be an important resource for the recognition of the cognitive state, medical disorders, and a better understanding of the brain in general. In this study, we have compared 51 mother wavelets taken from 7 different wavelet families, which are applied to a Stationary Wavelet Transform (SWT) decomposition of an EEG signal. This process includes Haar, Symlets, Daubechies, Coiflets, Discrete Meyer, Biorthogonal, and reverse Biorthogonal wavelet families in extracting five different brainwave subbands for source localization. For this process, we used the Independent Component Analysis (ICA) for feature extraction followed by the Boundary Element Model (BEM) and the Equivalent Current Dipole (ECD) for the forward and inverse problem solutions. The evaluation results in investigating the optimal mother wavelet for source localization eventually identified the sym20 mother wavelet as the best choice followed by bior6.8 and coif5.

## 1. Introduction

Brain-Computer Interface (BCI) not only external permits controlling devices but also interacts using the environment by brain signals. EEG signals measurements over the motor cortex exhibit changes in power related to the movements or imaginations which are executed in motor tasks [1]. Changes declare decrease or increase of power in alpha (8 Hz–13 Hz) and beta (13 Hz–28 Hz) frequency bands from resting state to motor imagery task known as event related synchronization and desynchronization [2]. The necessity to communicate with the external world for locked-in state (LIS) patients made doctors and engineers motivated to develop a BCI technology for typing letters through brain commands. Research has been done around this area to ascertain the dream of typing for the handicapped. In the brain, some regions of the cerebral cortex are involved in the planning, control, and execution of voluntary movements. Electroencephalography (EEG) signals are electrical potentials generated by the nerve cells in the cerebral cortex. In order to execute motoric tasks, the EEG signals have appeared over the motor cortex [1].

To accurately study and analyze the human brain, electroencephalography (EEG) [1] is thought to be the optimal method that helps us advance in our quest due to the noninvasiveness and the low-cost factors. The electroencephalogram (EEG) is a recording of the electrical activity of the brain from the scalp. The recorded waveforms reflect the cortical electrical activity. In fact, the EEG provides access to human brain activities in 5 main frequency band packages presented in Table 1 [2]. The scientific trend shifted towards exploiting these frequency subbands and seeking the extraction of pure and noncontaminated signals instead of developing recording methods and other ways to express the signal.

The research community took an omnidirectional approach throughout the recent years to try to extract the human brain activities and access these five different frequency subbands. In this context, Murali et al. [3] used the recurrence quantification analysis (RQA) algorithm and an adaptive FIR filter for the EEG signal extraction. As for Singh, Vivek et al. [4], they compared using Finite Impulse Response (FIR) and Infinite Impulse Response (IIR) filters and confirmed the FIR success over RII regarding EEG signals. On the other hand, Nallamothu et al. [5] used a Nonlinear Least Mean square (LMS) adaptive filtering to remove artifacts from the EEG signal.

For their part, Tzimourta et al. [6, 7] used a Discrete Wavelet Transform (DWT) for feature extraction and Support Vector Machine (SVM) classification of Epileptic Seizures. Actually, our previous work [8] has proved the effectiveness of the Stationary Wavelet Transform (SWT) using Symlet 4 mother wavelet compared to FIR filters in feature extraction of the alpha and gamma band waves. Furthermore, Akkar and Jasim [9] proved that the Symlet 9 mother wavelet is the best wavelet from a set of 25 mother wavelet functions using the Packet Wavelet Transform (PWT). Condo and Efrén [10] compared 18 different mother wavelets for EEG signal analysis and affirmed Symlet 6 and Daubechie 5 are the most adequate for EEG signals. Noor et al. [11] compared 45 mother wavelets to conclude that Symlet 9 followed by Coiflet 3 and Daubechie 7 exhibits the highest similarities and compatibilities with the EEG signal after applying an FIR notch filter.

The EEG signal is a nonstationary signal; the advantage of using the wavelet transform over the usual Fourier transform in EEG signals is their capability to analyze nonstationary signals [12, 13] due to their improved presentation in both the time and frequency domain as shown by Figure 1.

In this context, this study aims at comparing 51 different mother wavelets using SWT to extract human brainwaves and localize their sources. In section 2, we will address the methodology first, by describing the manipulated dataset and then proceed by presenting the SWT and the processing steps of our study and finally by introducing the evaluation methods.  Section 3 will feature the conceived results and section 4 will highlight the discussion.

## 2. Methodology

### 2.1. Dataset

#### 2.1.1. Simulated Signal

Influenced by the morphology and the structure of actual EEG signals, we created a sinusoidal signal with oscillations of 400 ms on 800 ms time windows used in the evaluation process.

A sampling rate of 1000 Hz and an oscillation frequency of 3, 6, 10, 20, and 45 Hz were recorded for the extraction of Delta, Theta, Alpha, Beta, and Gamma waves, respectively. The signal to the noise ratio (SNR) was also altered from −5 to 15 dB with −5 dB for noisy signal simulation, 10 dB for balanced signals, and 15 dB for acceptable quality signals. On the other hand, the amplitude of the signal depends on both the SNR value and the noise contaminating the signal, which is what is known as a pink noise; besides, it is a very common noise for biological systems.

#### 2.1.2. The EEG Dataset

The EEG signal dataset used in this study is a one-subject recording of a presurgical EEG signal from a pharmacoresistant subject with asymptomatic focal cortical dysplasia in the right occipital-temporal junction. The acquisition and preprocessing phases were applied as in our previous work [7, 8] and validated by an expert neurologist. This particular EEG recording was chosen because it presented clear alpha and gamma patterns with regular spiking and visible epileptic oscillations as validated by the expert. The EEG data was recorded on a Deltamed System, with a 2500 Hz sampling rate and antialiasing low-pass analog filter set to 100 Hz. The dataset contained 74 epochs with a 6-second duration each, 62 channels, and 148 events.

### 2.2. The Wavelet Transform

Similar to the Fourier transform (FT), the wavelet transform (WT) is a function that grants the passage from the time to the frequency domain. However, the FT decomposes the signal into a series of sinus and cosines components as in the following equation:

(1) $$\begin{array}{c} s\left(t\right)=\int_{\omega =-\infty }^{+\infty }S\left(\omega \right)e^{j\omega t}\text{d}\omega , \end{array}$$

with S(*ω*) the short-time Fourier coefficient controlled using the frequency parameter *ω*.

The wavelet transform also decomposes the signal into a series of wavelet component as in the following equation:

(2) $$\begin{array}{c} s\left(t\right)=\int_{a=0}^{+\infty }\int_{b=0}^{+\infty }c\left(a,b\right)\varphi_{a,b}\left(t\right)\text{d}a.\text{d}b, \end{array}$$

where *C*(*a*, *b*) is the wavelet coefficient and *φ*_*a*,*b*_(*t*) the mother wavelet with “*a*” the scaling parameter and “*b*” the wavelet shifting parameter that determines the shape of the wavelet. In fact, Figure 2 highlights the difference between FT and WT decomposition components. Moreover, the wavelets are characterized by a limited duration, irregularity, and asymmetricity compared to the predictable, fluid, and infinitely propagated sinus waveform.

On the other hand, the wavelet transform used in this study is the stationary one (SWT) instead of the Continuous Wavelet Transform (CWT) or the Discrete Wavelet Transform (DWT). In fact, the SWT is more suitable for our case by avoiding the frequency band overlapping of CWT [14] and preserving the properties of the signal by averting the binary decimation process (downsampling) of DWT [15, 16].

### 2.3. Levels of Decomposition and Processing Steps

In order to decompose the EEG signal of our dataset that has 2500 Hz sampling rate to extract the five EEG frequency subbands, we had to reduce the signal to exactly 2048 Hz sampling rate; otherwise, these subbands would be extremely overlapping. In Figure 3, we display the decomposition of the resampled EEG signal. We notice here that, in our previous study [8], we have not resampled the signal as we extracted only the alpha and gamma waves that were far separated and did not cause band overlapping issues. Our decomposition level was 9 to acquire access to the delta wave frequencies while our previous work needed only 7 levels of decomposition to reach the alpha wave. We can also notice that, in our previous work, the approximated coefficients cAi included upper and lower levels (for alpha wave extraction, the cAi were 6, 7, 8 and cDi was 7), while for this study, we have included only the above upper levels for the cAi (for alpha wave extraction, the cAi were 6, 7 and cDi was 7). The most studied characteristic of EEG signals in accordance with alertness level is Power Spectral Density (PSD) of different brain waves: delta, theta, alpha, and beta.

As the wavelet decomposition phase is completed, we evaluate the mother wavelets used in this process and move on to the source localization.  Figure 4 shows the processing steps of this study.

### 2.4. The Evaluation Methods

#### 2.4.1. The Goodness of Fit (GOF)

The goodness of fit (GOF) is an evaluation method commonly used for physiological signals that adopt Pearson's chi-squared statistical test [17], which is the normalized sum of squared deviations that investigate the likelihood of an observed difference in the frequency distribution compared to the theoretical distribution as in the following equation:

(3) $$\begin{array}{c} \mathrm{GOF}\;=\;1\;–\;\left(\frac{{}_{\sum }^{r}\sum_{t=1}^{r}{\left(s\left(t\right)-s_{f}\left(t\right)\right)}^{2}}{\sum_{t=1}^{r}s{\left(t\right)}^{2}}\right), \end{array}$$

where *s*(*t*) is the theoretical power and *s*_*f*_(*t*) the power of the extracted signal that depends on the adopted mother wavelet.

#### 2.4.2. The Power Spectral Density (PSD) and Scalp Topographies

The Power Spectral Density is a display of the data energy distribution throughout the frequency spectrum. It is used as a visual evaluation process for its efficiency in presenting the data in the frequency domain rather than the time domain, which allows the identification of the extracted EEG frequency bands [18]. The energy frequency distribution of the EEG signal channels compares the mother wavelets effectiveness in isolating the extracted frequency band from the other subbands or artifacts and differentiates its capabilities to amplify the extracted signal power.

On the other hand, the scalp topographies are another visual evaluation process since it represents a mapping of the brain activities distributed on the surface of the scalp. An increasingly dipolar topography suggests that a cerebral measurement is an observation of a discharge operation involving a big number of neurons. Even in nonepileptic observations of brain activities, the dipolar scalp topographies are a great indicator of a valuable recording session since they reflect the domination of certain areas over others in the energetic exertion, which is the typical and more natural habit of cerebral behavior [19].

#### 2.4.3. The Source Localization

The source localization is an estimation of the brain activity generator locations [20]. To reach this estimation, first, we solve the forward problem, which is a calculation of the field generated by a given source for an estimated brain shape and conductivity, with a consideration of numerous properties, such as the shape of the brain that changes from a subject to another or the anisotropy conductivity of the skull and the brain conductivity [21]. For the forward problem, we used the Boundary Element Model (BEM), which is a surface mesh calculation of interfaces between the tissues using the MRI of the patient (which makes it a realistic model) [22]. For the inverse problem, which is an estimation of the current generator distribution responsible for the electric EEG signal, we used the Equivalent Current Dipole (ECD), which is the most used method to simplify the brain activities in a few sources [23]. The signals are assumed to be generated by a small number of focal sources modeled by current dipoles (an unknown position, amplitude, and orientation). Moreover, the extracted signal has to undergo an independent component analysis (ICA) dipole fitting operation as a preprocessing phase before the ECD inverse problem solution, in order to separate different components and make the components in a dipolar state useful in the localization of the source generators. The ICA is the feature extraction phase compatible with the statistically independent and non-Gaussian signals, which are the traits of the EEG signal [24] while the ECD and the BEM are our classification algorithm [25].

In fact, the source localization process is sensitive to the quality of the extracted EEG frequency band and can also serve as an evaluation process that depends on the number of the located sources and the accuracy of their localization.

## 3. Results

### 3.1. The GOF Evaluation Results

The goodness of fit (GOF) is the evaluation process that enabled us to minimize both our wavelet selection and processing criteria. Considering that the other evaluation methods and the source localization are a computationally heavy and costly process, the GOF is an excellent fast evaluation that relieved us from repeating the hull processing steps and source localization for the vast number of 51 mother wavelets.  Figure 5 presents the GOF results for the 51 mother wavelets with different SNR values of −5, 10, and 15 dB as we have mentioned in the dataset descriptions in Section 2, A, 1).

On the other hand, the use of alpha and gamma wave extraction in GOF evaluation is justified by our earlier knowledge during our previous study [8] of the excellent capability of SWT in extracting these specific frequency subbands.

The GOF results showed a similar pattern across the different frequency subbands and different SNR values with a distinct superiority to sym20, coif5, bior6.8, rbio6.8, and dmey wavelets.

In order to explore and investigate this superiority, we have extracted the best mother wavelets of every wavelet family and the wavelets that already showed some noteworthy results in other studies, such as sym4 in [8], db5, and sym6 in [10] and sym9 in [9, 11], in every EEG frequency subband, as shown in Figure 6.

Besides, after isolating the GOF results about the limited number of noteworthy wavelets, we notice that the performance of the wavelet extraction changes from one frequency subband to another with an obvious preeminence in gamma and alpha waves. We also observe that sym4 in [8] is the lowest in the GOF performance due to the approximated coefficient choice in the decomposition phase compared to our choice of approximated coefficient in this study for all the wavelets.

Finally, to lock the GOF evaluation results, we calculated the noteworthy wavelet average across the five frequency subbands and ordered them from the lowest performance, on the left, to the best performance, on the right by their GOF score in Figure 7. In fact, the best results were achieved using demy and sym20 wavelets, while the worst results used sym4 [8] and Haar also.

### 3.2. The PSD and Topographies Evaluation Results

The Power Spectral Density (PSD) is also an important evaluation method that grants us a visual representation of the EEG signal extraction. The choice of frequency subband extraction visualization for this evaluation was limited to the alpha and gamma waves for the confirmed potential of SWT in their extraction. Moreover, due to the weak energy of the gamma wave and its proximity to the 50 Hz noise artifact of the original EEG signal dataset, we relied only on the alpha wave in the PSD visualization as it provides a clear display of the extraction effectiveness difference between the selected mother wavelets.

In Figure 8, we compare the EEG signal extraction of the alpha frequency subband using the different noteworthy wavelets chosen by the GOF evaluation ordered from the worst to the best. As we can deduce, the haar and sym4 wavelets, respectively, had the worst results with a signal spectrum contaminated by different artifacts and other frequency subbands while sym20 and dmey had the best results in isolating the extracted signals from other infiltrating ones. We can also recognize the abilities of the new SWT decomposition in eliminating high frequency, while witnessing some difficulties in low-frequency elimination, such as delta and theta, as demonstrated in the PSD visualization.

For the scalp topography visualization, almost all the noteworthy mother wavelets selected by the GOF had similar good results by producing depolarized scalp topographies isolated from the other frequencies, except for the Haar and sym4 wavelet extractions, which produced some interfering artifacts that could compromise the ability to review the scalp topographies by the medical experts and mislead them in diagnosing the cause of these parasites.  Figure 9 displays the scalp topographies of the original signal compared to both the mother wavelet extraction and the contaminated scalp topographies of Haar and sym4. As an assessment of the PSD and scalp topography evaluation, the sym20 and demy mother wavelets demonstrated the best results while the Haar and sym4 produced the worst ones.

### 3.3. The Source Localization

For the source localization, we performed the Independent Component Analysis (ICA) on the extracted signals by the noteworthy mother wavelets; then, we used the BEM for the forward problem and ECD for the inverse problem. As we have already mentioned, the ICA is a computationally costly process for feature extraction, especially with 62 EEG channels for the extraction of the same number of components before the source localization, so we reduced the process to include only the alpha and gamma frequency subbands. The alpha wave is the most important brainwave activity in the human brain and the gamma wave is perceived as an indicator of high active cognitive state and constantly used in brain malfunction and disease confirmation [26].

The ICA was performed using the runica algorithm from the EEGLAB toolbox [27]. Then, the BEM and ECD were executed using the fieldtrip toolbox [28]. We set a rejection threshold for the components based on the Residue Variance equivalent to RV = 15% as it is the optimum value in component rejection, as confirmed by Artoni et al. [29]. In Figure 10, we present the source localization of the alpha and gamma extracted waves using the different noteworthy mother wavelets. As we can see, every mother wavelet extraction has a different number of sources localized under the Residue Variance (RV) error threshold and different source locations compared to each other. In order to evaluate the source localization of our different mother wavelets, we focus on the number of localized components by every mother wavelet and the number of times every mother wavelet has the best accuracy (lower RV value) in localizing the source of a component and the average of accuracy in the five first components. The reason for which we have included the accuracy of the five first components in our evaluation is that the ICA using the runica algorithm for the output components in a decreasing order of the EEG variance accounted for by each component, that is, the lower the order of a component, the more data (neural and/or artifactual) it accounts for [30].

Figure 11 shows the number of components localized by each mother wavelet in the alpha and gamma frequency subbands and only the number of components that were not localized in the other frequency subbands.

An interpretation of the number of localized component results showed that the sym20 mother wavelets produced the best results followed by Haar and bior6.8, while coif5 had the lowest number of localized components.

In Figure 12, we explore the accuracy of the noteworthy mother wavelets in source localization by comparing the number of times each mother wavelet managed to record the lowest RV score. This chart also considers the localization in the alpha wave, gamma wave, and the combined best-localized components of both frequency subbands.

The sym20 mother wavelet scored the best accuracy results followed by Haar and sym9, while rbio 6.8 did not have even once the best accuracy compared to the other wavelets for both frequency subbands. We also spot that the original EEG signal had an impressive accuracy in gamma wave, which indicates the interference of the other frequency subbands or the 50 Hz noise artifact and compromised the integrity of the located sources considering that the gamma wave had poor frequency energy that could not produce such result.

Table 2 presents the final criteria for source localization evaluation that focuses on the accuracy of the five first components. The accuracy is expressed with the RV values, which means that the lower the RV value is, the better accuracy will be.

Actually, the best result for the alpha wave was achieved by bior6.8 while the worst was recorded by the Haar mother wavelet. For the gamma wave, the Haar mother wavelet produced the best result, while rbio6.8 extractions were last compared to the other wavelet extractions. Then, regarding the combined best-localized components of alpha and gamma, the sym20 and coif5 shared the first place in extracting the most accurate first five components, with the rbio6.8 mother wavelet in the last place.

As an overall perception of the source localization results in evaluating our mother wavelets, we can classify the sym20 mother wavelet as the best mother wavelet extraction overall, while the Haar occupies the second place with questionable results due to our previous readings of the GOF, PSD, and scalp topographies that proved the interference of frequency overlapping and noise artifacts in the sincerity of the localized components. If we eliminate the Haar mother wavelet, we must crown the bior6.8 mother wavelet the second place considering the number of localized components and the best results achieved in the accuracy average of the first components in the alpha wave followed by the coif5 and sym9 mother wavelets. While On the other hand, the dmey produced a somehow moderate result in light of the promising potential in the earlier evaluations of GOF, PSD, and scalp topographies. The least favorite mother wavelet in source localization was the rbio6.8 with the worst accuracy results recorded by all the noteworthy mother wavelets.

## 4. Conclusion

In this paper, we have compared 51 different mother wavelets taken from 7 different families including Haar, Symlets, Daubechies, Coiflets, Discrete Meyer, Biorthogonal, and reverse Biorthogonal, which are applied to source localization and extraction of EEG signal. For the source localization performance comparison, the 10 mother wavelets selected from the 51 mother wavelets produced an adequate result. However, the sym20 outshined all the other wavelets and took the lead almost in every evaluation followed by a notable performance from bior6.8, coif5, and sym9, respectively. Then, the least results were produced by the Haar and rbio6.8 mother wavelets. As a conclusion, the Symlet family generates the top results for EEG signal, as demonstrated by our study. Then, bior6.8 and coif5 are the second important mother wavelets for source localization.

Regarding the evaluation methods, we used the goodness of fit (GOF), the Power Spectral Density, and scalp topographies in the extraction of EEG frequency subbands applied to benchmarks containing source localization with the number of located sources and accuracy of localization. The source localization is produced via Stationary Wavelet Transform (SWT) and an Independent Component Analysis (ICA) feature extraction followed by Boundary Element Model (BEM) and Equivalent Current Dipole (ECD) solutions for the forward and inverse problem. Future studies and advancements could explore the improvement of the source localization feature extraction or forward and inverse problem solutions. The use of artificial intelligence techniques based on the deep neural network could help to facilitate the simulation and give better results.

## Figures and Tables

**Figure 1:** Comparison between the partition of Fourier transform and wavelet transform in the time-frequency domain. (a) Fourier transform. (b) Wavelet transform.

**Figure 2:** Comparison between (a) FT decomposition component and different mother wavelets families decomposition components. (b) Symlets 4 (c) Coiflets 5. (d) Daubechies 11.

**Figure 3:** EEG signal SWT decomposition levels with cAi as the approximated coefficients and cDi as the detailed coefficients.

**Figure 4:** The cycle of processing steps during this study.

**Figure 5:** The GOF results in alpha and gamma waves with 51 mother wavelets using SNR values of −5, 10, and 15 dB.

**Figure 6:** The results of the average GOF for every EEG frequency subband with the selected mother wavelets across the SNR values of −5, 10, and 15 dB.

**Figure 7:** The GOF average of the noteworthy wavelets across the EEG frequency subbands and SNR values ranked from left to right by order of best performance.

**Figure 8:** PSD visualization of the different noteworthy mother wavelets in alpha wave extraction.

**Figure 9:** A scalp topographies comparison between the original dataset, the noteworthy mother wavelets extractions, and the contaminated scalp topographies of Haar and sym4 wavelets for the five EEG frequencies subbands.

**Figure 10:** Visualization of the alpha and gamma waves source localization using the noteworthy mother wavelets extractions.

**Figure 11:** The number of components localized by the noteworthy mother wavelets in alpha and gamma waves with RV under 15%.

**Figure 12:** The number of times each mother wavelet scored the best accuracy for source localization in alpha and gamma waves.

**Table 1:** The EEG signal main human brain frequencies.

EEG bands		Frequency (Hz)	Main description
Delta		0–4	Deep state of sleep
Theta		4–8	Deep meditation and lucid dreaming
Alpha		8–12	Relaxation/creativity
Beta		12–32	Analytical thinking or stress/anxiety
Gamma	Lower	32–64	Wide brain activities or higher 64–128 brain disorder
	Higher	64–128	

**Table 2:** The RV average of 5 first components for the noteworthy mother wavelets.

Wavelet	Alpha RV average of 5 first components	Gamma RV average of 5 first components	Combined RV average of best 5 first components
Original dataset	10.8		
Sym4	8.9	9.5	8.6
Sym6	7.8	9.6	7.7
Sym9	6.8	10.2	6.8
Sym20	9.4	9.6	6.2
Haar	10.9	8.3	6.7
Db5	7.8	9.7	7.8
Coif5	8.8	10.2	6.2
Bior6.8	6.7	9.6	6.6
Rbio6.8	9.3	10.4	9.3
demy	9.4	9.6	6.8

## Data Availability

The medical used data are available from the corresponding author upon request.

## References

[1] Berger H. (1929). Über das elektrenkephalogramm des menschen. *Archiv für Psychiatrie und Nervenkrankheiten*.

[2] Sanei S. (2013). *Adaptive Processing of Brain Signals*.

[3] Murali L., Chitra D., Manigandan T., Sharanya B. (2016). An efficient adaptive filter architecture for improving the seizure detection in EEG signal. *Circuits, Systems, and Signal Processing*.

[4] Singh V., Veer K., Sharma R., Kumar S. (2016). Comparative study of FIR and IIR filters for the removal of 50 Hz noise from EEG signal. *International Journal of Biomedical Engineering and Technology*.

[5] Nallamothu S. S., Dodda R. K., Dasara K. S. (2018). *Eye Blink Artefact Cancellation in EEG Signal Using Sign-Based Nonlinear Adaptive Filtering Techniques. Information Systems Design and Intelligent Applications*.

[6] Tzimourta K. D. (2018). *Epileptic Seizures Classification Based on Long-Term EEG Signal Wavelet Analysis. Precision Medicine Powered by Health and Connected Health*.

[7] Kandilli C., Mertoglu B. (2020). Optimisation design and operation parameters of a photovoltaic thermal system integrated with natural zeolite. *International Journal of Hydromechatronics*.

[8] Abdennour N. Extraction and localization of non-contaminated alpha and gamma oscillations from EEG signal using finite impulse response, stationary wavelet transform, and custom FIR.

[9] Akkar A. H., Jasim F. A. (2017). Optimal mother wavelet function for EEG signal analyze based on packet wavelet transform. *International Journal of Scientific & Engineering Research*.

[10] Condo L., Efrén L. Comparison of wavelet transform symlets (2–10) and daubechies (2–10) for an electroencephalographic signal analysis.

[11] Noor A.-Q. (2015). Selection of mother wavelet functions for multi-channel EEG signal analysis during a working memory task. *Sensors*.

[12] Trimeche K. (2019). *Generalized Wavelets and Hypergroups*.

[13] Safa M., Ahmadi M., Mehrmashadi J. (2020). Sedghi Selection of the most influential parameters on vectorial crystal growth of highly oriented vertically aligned carbon nanotubes by adaptive neuro-fuzzy technique. *International Journal of Hydromechatronics*.

[14] Rhif M., Ben Abbes A., Farah I., Martínez B., Sang Y. (2019). Wavelet transform application for/in non-stationary time-series analysis: a review. *Applied Sciences*.

[15] Wang S.-H., Zhang Y.-D., Dong Z., Phillips P. (2018). *Wavelet Families and Variants. Pathological Brain Detection*.

[16] Sedghi C., Yan W., Cai X., Liu S., Li T. H., Li G. (2020). Neural saliency algorithm guide bi-directional visual perception style transfer. *CAAI Transactions on Intelligence Technology*.

[17] Zhang X. (2016). Localizing percentages of interictal 18 F-fluorodeoxyglucose (FDG)-PET and magnetoencephalography (MEG) in pre-surgical evaluation of 107 consecutive patients with non-lesional epilepsy. *International Journal of Clinical & Experimental Medicine*.

[18] Petroff O. A., Spencer D. D., Goncharova I. I., Zaveri H. P. (2016). A comparison of the power spectral density of scalp EEG and subjacent electrocorticograms. *Clinical Neurophysiology*.

[19] Mammone N., Inuso G., La Foresta F., Versaci M., Morabito F. C. (2011). Clustering of entropy topography in epileptic electroencephalography. *Neural Computing and Applications*.

[20] Song J., Davey C., Poulsen C. (2015). EEG source localization: sensor density and head surface coverage. *Journal of Neuroscience Methods*.

[21] Azizollahi H., Aarabi A., Wallois F. (2016). Effects of uncertainty in head tissue conductivity and complexity on EEG forward modeling in neonates. *Human Brain Mapping*.

[22] Gaul L., Kögl M., Wagner M. (2013). *Boundary Element Methods for Engineers and Scientists: An Introductory Course with Advanced Topics*.

[23] Elaina N. S. Somatosensory source localization for the magnetoencephalography (MEG) inverse problem in patients with brain tumor biomedical Engineering (ICoBE).

[24] Du K.-L., Swamy M. N. S. (2014). *Independent Component Analysis. Neural Networks and Statistical Learning*.

[25] Ali Z., Mahmood T. (2020). Complex neutrosophic generalised dice similarity measures and their application to decision making. *CAAI Transactions on Intelligence Technology*.

[26] Hiroki N. (2017). Scalp EEG ictal gamma and beta activity during infantile spasms: evidence of focality. *Epilepsia*.

[27] Delorme A., Makeig S. (2004). EEGLAB: an open source toolbox for analysis of single-trial EEG dynamics including independent component analysis. *Journal of Neuroscience Methods*.

[28] Oostenveld R., Fries P., Maris E., Schoffelen J.-M. (2011). FieldTrip: open source software for advanced analysis of MEG, EEG, and invasive electrophysiological data. *Computational Intelligence and Neuroscience*.

[29] Artoni F., Menicucci D., Delorme A., Makeig S., Micera S. (2014). RELICA: a method for estimating the reliability of independent components. *NeuroImage*.

[30] Delorme A., Sejnowski T., Makeig S. (2007). Enhanced detection of artifacts in EEG data using higher-order statistics and independent component analysis. *Neuroimage*.

[31] Kaur M., Singh D. (2021). Multi-modality medical image fusion technique using multi-objective differential evolution based deep neural networks. *Journal of Ambient Intelligence and Humanized Computing*.

[32] Kaur M., Singh D. (2020). Fusion of medical images using deep belief networks. *Cluster Computing*.

[33] Murlidhar B. R., Sinha R. K., Mohamad E. T., Sonkar R., Khorami M. (2020). The effects of particle swarm optimisation and genetic algorithm on ANN results in predicting pile bearing capacity. *International Journal of Hydromechatronics*.

